This article has been retracted.

# Efficacy and Safety of Glycosides of Tripterygium wilfordii Combined with Renin-Angiotensin System in the Treatment of IgA Nephropathy: A Systematic Review and Meta-Analysis

**DOI:** 10.1155/2022/5314105

**Published:** 2022-09-30

**Authors:** Ming Chen, Peiqing Zhang, Lianhua Li, Zhuo Yu, Na Liu, Lifan Wang

**Affiliations:** Heilongjiang Academy of Traditional Chinese Medicine, Department of Nephropathy, Heilongjiang 150036, China

## Abstract

**Background:**

IgA nephropathy (IgAN) is currently the most common primary glomerular disease, accounting for approximately 36.7% to 58.2% of primary glomerular disease in kidney biopsies in China. Definitive diagnosis depends on immunopathological examination of the kidney. The prognosis of this disease was generally considered to be good, but recent studies have found that about half of patients can progress to end-stage renal disease within 30 years of onset. Because the pathogenesis is unknown, there is no specific treatment.

**Objective:**

To evaluate the efficacy and safety of glycosides of Tripterygium wilfordii (GTW) in combination with renin-angiotensin system (RAS) inhibitors for the treatment of IgAN.

**Methods:**

Search Embase, Pubmed, Cochrane, CNKI, Web of Science, Wanfang, and VIP for all randomized controlled trials (RCTs) on treating IgAN with RASI from the self-built database to December 2021. Relevant data were searched and collected separately by two reviewers. The Cochrane risk of bias model was used for quality assessment, and RevMan 5.3 was used for data analysis.

**Results:**

Thirteen Chinese publications with a total of 958 patients were finally included. There was no statistically significant difference in baseline information (including laboratory data and clinical parameters) between the two groups of patients. The urine protein quantification in both groups showed a significant decreasing trend as the treatment duration increased. At 3, 6, 9, and 12 months after treatment, urine protein was significantly lower than the baseline value in both the observation and control groups (*P* < 0.05). During the follow-up period, there was no statistical difference in blood creatinine (Scr) and eGFR values between the two groups compared with the baseline values (*P* > 0.05). Patients with CKD stage 2 achieved a higher remission rate compared with patients with CKD stage 3, with a statistically significant difference (*P* < 0.05), and the difference between the two groups was not significant for patients in the same stage. There was no statistically significant difference in the total effective rate between the two groups (*P* > 0.05). During the follow-up period, there was no statistically significant difference in urine protein quantification, Scr, and eGFR between the two groups. In terms of the incidence of adverse reactions, the observation group was less than the control group, and there was a significant difference between the two groups (*P* < 0.05).

**Conclusion:**

GTW combined with RASI is one of the safe and effective treatment modes for IgAN nephropathy. It can not only effectively reduce the excretion of urinary protein in patients and delay the progression of chronic kidney disease but also has less serious side effects and is well tolerated by patients, so it can be a new choice of therapeutic drugs for this group of patients.

## 1. Introduction

IgA nephropathy (IgAN), also known as Berger's disease, is divided into two categories: primary and secondary. Primary IgA nephropathy is more common, accounting for about 36.7% to 58.2% of primary glomerular diseases diagnosed by renal pathology in China, and its incidence has been gradually increasing in recent years [1, 2]. It can be seen at any age, and patients aged 16–35 years account for about 80% of the total number of patients with the disease [3, 4]. The main pathological manifestation is the deposition of IgA-based immune complexes with or without IgG and IgM in the glomerular thylakoid region or capillary loops.

In terms of clinical manifestations, IgA nephropathy is characterized by varying degrees of hematuria, proteinuria, edema, hypertension, renal insufficiency, and, in a small number of patients, acute kidney injury (AKI) [5, 6]. The prognosis of this disease was generally considered to be good, but recent studies have shown that IgA nephropathy has a poor long-term prognosis and is one of the more important primary causes of end-stage renal disease (ESRD) in China. About 50% of patients progress to ESRD within 30 years and require renal replacement therapy to maintain life [7, 8]. The specific pathogenic effects and causative targets of IgA nephropathy remain unclear, and because its clinical manifestations vary and the severity of the disease varies, there are no uniform and standardized therapeutic measures, and most existing treatment regimens are centered on controlling risk factors [9, 10]. Persistent proteinuria >1 g/d, persistent severe hypertension, and renal impairment are the more important risk factors in the clinical manifestations of IgA nephropathy [11, 12]. The current treatment focuses on reducing proteinuria, controlling blood pressure levels, and slowing the progression of renal function.

The renin-angiotensin system (RAS) blockers are the most widely used drugs with proven efficacy in the treatment of IgA nephropathy, mainly including angiotensin-converting enzyme inhibitors (ACEI) and angiotensin II receptor antagonists (ARB). The 2012 KDIGO guidelines recommend long-term treatment with RAS blockers for patients with urine protein >1 g/d; RAS blockers are recommended for patients with urine protein between 0.5 and 1 g/d [13, 14].

Glycosides of Tripterygium wilfordii (GTW), an active ingredient extracted from the peeled root of Tripterygium wilfordii, is the most widely used Chinese patent immunosuppressant with powerful anti-inflammatory and immunosuppressive effects and is used more frequently in diabetic nephropathy and rheumatic diseases. Studies have shown [15, 16] that the most important active component of rehmannia polysaccharide, rehmannia lactone alcohol, significantly reduced serum IgA levels and improved abnormal IgA glycosylation in rats with IgA nephropathy. It has been shown to be effective in IgA nephropathy with normal renal function and moderate proteinuria, but its use in the treatment of IgA nephropathy with decompensated renal function has been less studied. Patients with abnormal renal function at the time of renal biopsy have more severe pathological damage and higher pathological grade, and they often show insensitivity to hormones. Therefore, in this study, we investigated the clinical efficacy of tretinoin combined with the RAS blocker by comparing it with glucocorticoid combined with the RAS blocker and explored the effectiveness and safety of tretinoin in reducing urinary protein and delaying the progression of chronic kidney disease so as to provide a theoretical basis for the clinical treatment of patients with IgA nephropathy.

## 2. Materials and Methods

### 2.1. Inclusion and Exclusion Criteria

#### 2.1.1. Inclusion Criteria

1. Studies should be published RCTs of GTWplus RASI in treating IgAN
2. Follow-up time is more than 3 months
3. IgAN diagnosis by renal biopsy
4. Complete data
5. The language of literature is limited to Chinese and English

#### 2.1.2. Exclusion Criteria

1. Non-RCT studies
2. Incomplete data
3. Failure to exclude patients with systemic diseases

### 2.2. Literature Search

By searching Embase, PubMed, Cochrane, CNKI, Web of Science, Wanfang, and VIP, the search interval was from the creation of the database to December 2021. Search terms were as follows: (“IgA nephropathy” or “glomerulonephritis, IgA”) and (“Tripterygium,” “Glycosides of Tripterygium wilfordii,” or “GTW”) and (“ACEI,” or “ARB,” “Puri,” or “Sartan,” or “RAS inhibitor”). Search for possible study titles, abstracts, and full text has been conducted.

### 2.3. Quality Assessment

Publication quality was evaluated according to the Cochrane risk of bias method. Two reviewers independently extracted data, evaluated the search results, and evaluated the full text when necessary, using standard data extraction methods for extraction. A third evaluator was asked to help resolve disagreement.

### 2.4. Data Collection and Analysis

Data such as participant characteristics, study baseline, and intervention characteristics for each group were extracted from all the included studies. The main results included complete remission (CR), partial remission (PR), and total remission (TR); UTP, Scr, and ALB were used as observation metrics; adverse events (AEs) were used as safety metrics. At least one of the above indicators is satisfying. Statistical analysis was performed using Cochrane RevMan 5.3. The heterogeneity between the literature is low (*P* ≥ 0.10; *I*^2^ ≤ 50%), and the heterogeneity is good; the fixed-effects model is used; the heterogeneity between the literature is poor (*P* < 0.10; *I*^2^>50%); a random-effects model is adopted; categorical variables choose odds ratio (OR) as the effect size, and continuous variables choose mean difference (MD) as the effect size, and the results are represented by forest plots. *P* < 0.05 is designated as significant.

### 2.5. Statistical Methods

SPSS 18.0 was used for analysis. The measurement data were described as the mean ± standard deviation $\left(\bar{x}\pm s\right)$ (normal data) or *M* (1/4, 3/4) (non-normal data); the count data were expressed as a number of cases and percentages. Quantitative data were compared using a *t*-test, and repeated measures data were analyzed by ANOVA for repeated measures; count data were compared using the *χ*^2^ test or rank sum test. Differences were considered statistically significant at *P* < 0.05.

## 3. Results

### 3.1. Literature Search and Screening Results

According to our criteria, we retrieved a total of 149 pieces of literature that met the requirements, all of them in Chinese; 54 pieces of literature were deleted, 67 pieces of literature were excluded from reading titles and abstracts, and 15 pieces of literature were excluded after reading the full text and finally included in this research literature 13 Article [10–22]; a total of 958 cases were included in this systematic review, including 431 cases in the treatment group and 527 cases in the control group. The retrieval process is shown in Figure 1, and the clinical data included in the literature are shown in Table 1.

### 3.2. Risk of Bias Assessment

Seven studies [12–14, 16, 18, 20, 21] mentioned a randomized design, one study [12] described allocation concealment, and one study [22] described a blinded design. None of the studies mentioned detection bias, except for 3 studies [14, 20, 21] that described complete outcome data, and 4 studies [14, 18, 20, 21] published incomplete outcome data. We performed a Cochrane risk of bias assessment, “+” low risk of bias, “−” high risk of bias, and “?” risk of bias is unknown. See Figures 2 and 3 for details.

### 3.3. TR

Among the 13 included studies, the definitions of TR, CR, and PR are different, as detailed in Table 2. The 5 studies [12–14, 17, 18] (the control group selected RASI as the treatment drug) compared the TR after 3 months of treatment, and the differences between the study groups were of little statistical heterogeneity (*P* = 0.97, *I*^2^ = 0%); a fixed-effects model was adopted. Data indicated that treatment TR was significantly better than control TR (OR = 4.3, 95% CI: 2.59, 7.16, *P* < 0.00001). 6 studies [10, 11, 15, 16, 21, 22] compared the TR after 6 months of treatment, and the statistical heterogeneity among the study groups was less (*P* = 0.97, *I*^2^ = 0%), and a fixed-effects model was adopted. Data indicated that treatment TR was significantly better than control TR (OR = 4.7, 95% CI: 2.77, 7.98, *P* < 0.00001). The subgroup analysis of the TR of the 3-month and 6-month treatment revealed less heterogeneity (*P* = 1.0, *I*^2^ = 0%), and a fixed-effects model was adopted. Data indicated no difference in the TR (OR = 4.49, 95% CI: 3.11, 6.48, *P* = 0.81) as shown in Figure 4. 3 studies [12, 14, 17] (the control group selected GTW as the treatment drug) with the TR after 3 months of treatment, and there was very little heterogeneity (*P* = 0.65, *I*^2^ = 0%), and a fixed-effects model was adopted. Data indicated that the treatment TR group was significantly better than the control TR group (OR = 3.85, 95% CI: 2.13, 6.97, *P* < 0.00001) as shown in Figure 5.

### 3.4. UTP

6 studies [12–14, 17–20] compared the quantitative changes of UTP in patients after 3 months of treatment. There was statistical heterogeneity (*P* < 0.0001, *I*^2^ = 83%), and no source accounting for it was found. Random effect model analysis revealed that treatments were significantly better controls (MD = −258.21, 95% CI: −358.67, −157.75, *P* < 0.00001). 5 studies [10, 11, 15, 16, 21] compared the quantitative changes of UTP after 6 months of treatment, and very little heterogeneity was found (*P* = 0.59, *I*^2^ = 0%), and fixed-effect model analysis revealed that treatments were significantly better controls(MD = −338.55, 95% CI: −431.63, −245.48, *P* < 0.00001). The UTP changes in the 3-month and 6-month treatment groups were analyzed by subgroup, and there was statistical heterogeneity among the study groups (MD = −338.55, 95% CI: −431.63, −245.48, *P* < 0.00001), and no source of heterogeneity was found. The random-effects model analysis revealed no difference (MD = −284.28, 95% CI: −365.94, −202.61, *P* = 0.25) as shown in Figure 6.

### 3.5. ALB

3 studies [13, 17, 18] compared the changes in ALB after 3 months of treatment and found heterogeneity among groups (*P* < 0.00001, *I*^2^ = 93%), and no source of heterogeneity was found. Random-effect model analysis revealed that ALB improvement in treatments was better than controls (MD = 5.04, 95% CI: 0.58, 9.5, *P* = 0.03). 4 studies [10, 11, 15, 16] compared the changes in ALB of patients after 6 months of treatment and found no heterogeneity (*P* = 0.0004, *I*^2^ = 83%), and the random-effect model analysis revealed no difference in ALB (MD = 1.26, 95% CI: 1.05, 3.57, *P* = 0.29). Subgroup analysis was performed on the ALB in the 3-month and 6-month treatment groups. There was statistical heterogeneity among the study groups (*P* < 0.00001, *I*^2^ = 93%), and random-effects model analysis demonstrated no difference in ALB (MD = 2.96, 95% CI: 0.29, 5.64, *P* = 0.14) as shown in Figure 7.

### 3.6. Scr

5 studies [13, 17–20] compared the changes in Scr of patients after 3 months of treatment and found heterogeneity among groups (*P* = 0.0003, *I*^2^ = 80%). Random-effect model analysis found that treatments improved Scr (MD = −5.07, 95% CI: −9.12, −1.01, *P* = 0.01); 4 studies [10, 11, 16, 21] compared the change in Scr after 6 months of the treatment. Results indicated heterogeneity among groups (*P* = 0.0009, *I*^2^ = 74%). Random effect model analysis found that treatments improved Scr (MD = −6.92, 95% CI: −10.73, −3.10, *P* = 0.02). Subgroup analysis was performed on Scr in the monthly group. There was statistical heterogeneity among the study groups (*P* < 0.00001, *I*^2^ = 79%). Random effect model analysis found no difference in Scr (MD = −6.92, 95% CI: −10.73, −3.10, *P* = 0.3) as shown in Figure 8.

### 3.7. AE

Among the included studies, 5 studies did not mention the occurrence of AE, and AEs were reported in the other 8 studies (Table 3), all of which described that the AEs were relieved and controlled after effective treatment, and there were no withdrawals due to AE. We compared the incidence of AE among the 8 included studies, of which 4 studies [12, 13, 17, 18] compared the incidence of AE after 3 months of treatment and found little heterogeneity (*P* = 0.20, *I*^2^ = 35%); fixed-effect model analysis revealed a significant difference in AE incidence between the groups (OR = 2.01, 95% CI: 0.79, 5.11, *P* = 0.14). 4 studies [10, 11, 15, 22] compared the occurrence of AE after 6 months of treatment, and there was little statistical heterogeneity among the groups(*P* = 0.48, *I*^2^ = 0%); the fixed-effect model analysis revealed that 6-month treatment drastically increased AE (OR = 2.31, 95% CI: 1.15, 4.66, *P* = 0.02). The subgroup analysis of AE in the 3-month and 6-month treatment groups showed very little heterogeneity (*P* = 0.48, *I*^2^ = 0%), and the fixed-effect model analysis revealed no difference in AE (OR = 2.20, 95% CI: 1.26, 3.85, *P* = 0.82) (Figure 9).

### 3.8. Publication Bias Assessment

Taking the TR as an example, a funnel plot was drawn to detect whether there was a small sample size publication bias. The results indicated that the studies were basically distributed on two sides of the funnel plot line. It can be clearly observed that the included literature has a certain degree of skewed distribution. The risk of publication bias is low (Figure 10).

## 4. Discussion

IgA nephropathy is currently the most prevalent primary glomerular disease in China [17, 18]. Patients with ESRD can only rely on hemodialysis, peritoneal dialysis, or renal transplantation to maintain their lives, and the quality of life of patients and their families is significantly reduced. Therefore, it is necessary to treat IgA nephropathy through active and effective measures to reduce urinary protein and slow down the progression of renal function. A number of studies have been conducted to investigate the factors affecting the prognosis of IgA nephropathy. Analyses have shown that patients with persistent large amounts of proteinuria, persistent uncontrolled hypertension, and renal impairment at the onset of disease have relatively severe renal pathology, poor long-term prognosis, and relatively poorer response to medications [21–23].

The duration of urinary protein has a greater impact on renal prognosis than the amount of urinary protein. Studies [24, 25] found that patients with urine protein >3 g/d had 25 times faster decline in renal function compared to patients with urine protein quantification <1 g/d. When urine protein decreased to less than 1 g/d in patients with massive proteinuria, the rate of decline in renal function slowed, and the natural course of the disease was similar to that of patients with low urine protein. Patients with urine protein less than 0.5 g/d have a better long-term prognosis than those with urine protein between 0.5 and 1 g/d. Studies [7, 26] have observed the natural course of IgA nephropathy and found that GFR decreases at an average rate of 1 to 3 ml/min per year in patients with normal renal function at presentation, while it increases rapidly to 9 ml/min per year in those presenting with nephrotic syndrome. The state of renal function at presentation also reflects the severity of pathological damage. Patients with renal insufficiency have a relatively high degree of thylakoid hyperplasia, a higher proportion of glomerulosclerosis, and often a higher Lee's classification [27, 28]. As the eGFR decreases and the residual glomeruli decrease, the rate of eGFR decline is accelerated, and once the blood creatinine exceeds 265.2 umol/L, the rate of GFR decline can reach 20 ml/min per year [29, 30]. Therefore, although the blood creatinine of patients in CKD2-3 is relatively not high, the renal impairment will be further aggravated if timely treatment is not carried out, and the CKD2-3 stage is also the last time for effective intervention before patients enter ESRD [31, 32].

Although the pathogenesis of immune complex deposition in glomeruli due to abnormal body immunity is widely recognized, opinions differ on whether immunosuppressive agents should be used alone or in combination in the treatment of IgA nephropathy [33, 34]. The 2012 KDIGO guidelines recommend 6 months of glucocorticoid therapy for patients with GFR >50 ml/min and persistent urinary protein >1 g/d despite 3–6 months of supportive therapy [35, 36]. However, no treatment recommendations are available for patients with proteinuria, GFR <50 ml/min, and not in ESRD. The incidence of autoimmune diseases has been increasing in recent years, and with it, the use of glucocorticoids has become more widespread [37]. The abuse of glucocorticoids has been accompanied by adverse effects of hormones such as femoral head necrosis, diabetes mellitus, and severe fatal infections, making the overall cost of the disease higher, and some patients are unable to tolerate them, refusing to take them, and easily giving up treatment and increasing the risk of disease progression.

Since the 1970s, when the effectiveness of tretinoin application in nephritis was demonstrated, various tretinoin products have been gradually and widely used in the treatment of chronic glomerulonephritis [38]. With the improvement of the pharmaceutical process, the initial tretinoin tonics have been replaced by preparations such as tretinoin polysaccharide tablets, with a significant reduction in adverse effects. In previous studies, tretinoin polysaccharide was mainly used in patients with IgA nephropathy with normal renal function and related treatment regimens such as tretinoin alone or in double doses, tretinoin combined with RAS blockers, tretinoin combined with hormones, and mortification of mortification, all of which showed good effects in reducing urinary protein and delaying the progression of renal function [39]. The results of this study also confirmed the significant efficacy of raglan polysaccharide combined with RAS blockers with fewer adverse effects in patients with IgA nephropathy in CKD stages 2-3.

The mechanism of raglan polysaccharide in IgA nephropathy is (1) inhibition of proliferation of thylakoid cells and stroma: the basic change of IgA nephropathy is the proliferation of glomerular thylakoid cells and stroma due to the stimulation of immune complexes in the thylakoid region. Previous animal studies have shown that the most important monomer of tretinoin that exerts immunosuppressive and anti-inflammatory effects is tretinoin lactone alcohol. This component can significantly reduce the level of serum IgA in rats with IgA nephropathy and improve the degree of abnormal glycosylation, as well as downregulate the level of the CD71 molecule, the main receptor of IgA1 in the glomerular thylakoid region, and reduce the deposition of IgA1 in the thylakoid region, thus inhibiting the proliferation of glomerular thylakoid cells and the increase of stroma [40]; (2) protection of podocytes: raffinose polysaccharide can stabilize the podocyte skeleton, reduce the damage to the podocytes, and protect the podocytes. Protection of podocytes: raglan polysaccharide can stabilize the podocyte skeleton, reduce podocyte damage, and increase the expression of nephrin and podocin, the key molecules of podocyte surface lytic membrane; (3) improvement of the glomerular filtration barrier: it mainly includes the repair of mechanical and charge barriers, thus reducing the loss of urinary protein in patients; (4) anti-inflammation, inhibition of immune response, and reduction of glomerular damage by cytokines. Thus, raglan polysaccharide has a clinical and basic test-proven effect on repairing and ameliorating the pathological damage of IgA nephropathy, which can effectively slow down the natural course of the disease.

The stability of the renin-angiotensin system, or RAS system, is essential for maintaining normal renal physiological function. Abnormally glycosylated IgA1 deposited in the glomerular thylakoid region can specifically activate the local RAS system in the kidney, which is one of the important causes of the development of IgA nephropathy. Therefore, RAS blockers are well-proven effective drugs for the treatment of IgA nephropathy. In particular, RAS blockers are recommended for patients with urinary protein >0.5 g/d, regardless of whether blood pressure is elevated or not, when blood pressure is tolerated.

It can be seen that the feasibility and practicality of combining RAS blockers with raglan polysaccharides are high. Therefore, this study included patients with IgA nephropathy with eGFR between 30 and 90 ml/(min-1.73 m^2^) and investigated the efficacy and side effects of a regimen of regimen polysaccharide combined with RAS blocker in the treatment of IgA nephropathy patients with CKD stage 2 to 3 by comparing the commonly used classical drugs, i.e., hormones combined with RAS blockers so as to clarify the superiority of the regimen of regimen polysaccharide combined with the RAS blocker. The superiority of the regimen of regioidoside combined with the RAS blocker in treating these patients was clarified.

Based on the above, the effect of GTW combined with RASI on IgAN was evaluated, hoping to provide a scientific basis for IgAN treatment. This study conducted a meta-analysis by screening existing randomized controlled trial studies and found that GTW plus RASI for IgAN improved the TR of treatment, decreased the quantification of double colic, increased ALB, and improved renal function. Specific findings showed that GTW combined with RASI was superior to GTW or RASI alone after 3 months of treatment in terms of total clinical efficacy. After 6 months of GTW in combination with RASI, it had an advantage over RASI alone. There was no significant advantage compared to 3 months of treatment. In terms of double stranding, GTW combined with RASI for 3 and 6 months had an advantage compared to the RASI group alone, but there was no significant advantage in reducing double stranding compared to treatment for 6 and 3 months; in terms of alcoholic gonadal function antipulmonary function anti-inflammatory patients, GTW combined with RASI for 3 months had an advantage in improving ALB compared to the RASI group alone. There was no significant advantage of GTW combined with RASI treatment for 6 months in terms of improvement in ALB compared to RASI alone. There was no significant advantage compared to treatment at 6 months and 3 months. In terms of Scr, GTW combined with RASI at 3 and 6 months of treatment had an advantage in improving renal function compared with RASI alone, but there was no significant advantage in reducing renal function at 6 months of treatment and after 3 months of treatment; in terms of AE, there was no difference between GTW plus RASI at 3 months and RASI alone, but the incidence of adverse reactions at 6 months of treatment was higher than with RASI alone.

The results of this clinical trial showed that raglan polysaccharide combined with the RAS blocker not only reduced urinary protein but also delayed the progression of renal function and was a safe and effective treatment option for CKD stage 2 to 3 IgA nephropathy. The abnormal menstrual events that occurred during treatment mostly improved after discontinuation of the drug and had less impact on older patients. For the possible events of hematocrit and abnormal liver function, they can be avoided by only closely monitoring the changes in routine blood and liver function of patients.

## 5. Conclusion

1. For patients with chronic kidney disease IgA nephropathy, tretinoin polysaccharide combined with the RAS blocker can not only effectively control urinary protein but also delay the progression of renal function
2. The efficacy of tretinoin combined with the RAS blocker is remarkable, with few adverse effects and no serious side effects such as abnormal glucose and osteoporosis of glucocorticoids, which is significantly superior compared with hormones
3. Patients with different stages of chronic kidney disease respond differently to treatment, and those in lower stages have better responsiveness to treatment and are more likely to achieve clinical remission [41]

## Figures and Tables

**Figure 1:** Flowchart of the process for selecting studies for the systematic review.

**Figure 2:** Risk of bias graph.

**Figure 3:** Risk of bias summary. “+” low risk of bias, “−” high risk of bias, and “?” unclear risk of bias.

**Figure 4:** Comparison of GTW combined with RASI versus RASI TR-3 months versus 6 months.

**Figure 5:** Comparison of GTW combined with RASI versus GTWTR-3 months.

**Figure 6:** GTW combined with RASI versus control UTP-3 months versus 6 months.

**Figure 7:** Comparison of GTW combined with RASI versus control group ALB-3 months versus 6 months.

**Figure 8:** GTW combined with RASI versus control Scr-3 months versus 6 months.

**Figure 9:** GTW combined with RASI versus control AE-3 months versus 6 months.

**Figure 10:** Funnel plots of TR published bias.

**Table 1:** Characteristics of the studies included in this systematic review.

Studies	Baseline characteristics of participants	Interventions/Controls
Shen 2009	*N*: 52 Gender: M26 F26; Age: 32 .48 ± 10.12 (18–60); UTP: 1.0–3.5 g/d; Ccr > 60 ml/min; Pathology: WHO II (12), III (30), IV (10).	*I* (*n* = 26): GTW (1 mg/kg/d), Benazepril (10 mg/d). C (*n* = 26): benazepril (10 mg/d). Follow-up period: 6 months

Yu 2012	*N*42; Age: 37.10 ± 10.70; UTP: 1.0–3.5 g/d; Normal renal function.	*I* (*n* = 20): GTW (60 mg/d), fosinopril (10–20 mg/d). *C* (*n* = 22): fosinopril (10–20 mg/d). Follow-up period: 6 months.

Yang 2014	*N*96; Gender: *A*: M17 F14; *B*: M19 F14; C: M17 F15; Age: *A*: 49.3 ± 10.6; *B*: 51.1 ± 12.3; *C*: 50.01 ± 10.12; UTP: <1.0 g/d.	*A* (*n* = 31): benazepril (10 mg/d).*B* (*n* = 33): GTW (60 mg/d). *C* (*n* = 32): GTW (60 mg/d), benazepril (10 mg/d). Follow-up period: 3 months.

Xiang 2014	*N*60; Gender: *I*: M18 F12; *C*: M19 F11 Age: *I*: 50.3 ± 9.6; *C*: 51.3 ± 8.2; UTP: <3.5 g/d; normal renal function. Pathology: Lee II ∼ III.	*I* (*n* = 30): GTW (1 mg/kg/d), telmisartan (80 mg/d). *C* (*n* = 31): telmisartan (80 mg/d). Follow-up period: 3 months.

Yu 2016	*N*90; Gender: *I*: M15 F15; C1: M16 F14; C2: M14 F16; Age: *I*: 46.1 ± 9.4; *C*1: 45.2 ± 5.7; *C*2: 45.9 ± 4.1;	*I* (*n* = 30): GTW (60 mg/d), benazepril (10 mg/d).*C*1 (*n* = 30): benazepril (10 mg/d). *C*2 (*n* = 30): GTW (60 mg/d).Follow-up period: 3 months.

Zhu 2017	*N*60; Gender: *I*: M15 F15; *C*: M17 F13; Age: *I*: 39.5 ± 12.5; *C*: 34.9 ± 11.5; UTP: 1.0–3.5 g/d; Normal renal function.	*I* (*n* = 30): GTW (60 mg/d), ARB. *C* (*n* = 30): ARB. Follow-up period: 6 months.

Cai 2018 [16]	*N*68; Gender: *I*: M19 F15; *C*: M18 F16; Age: *I*: 46.12 ± 9.05; C: 45.78 ± 8.83; UTP: 1.0–3.5 g/d.	*I* (*n* = 34): GTW (60 mg/d), telmisartan (40–80 mg/d). *C* (*n* = 34): telmisartan (40–80 mg/d). Follow-up period: 6 months.

Liang et al. 2019 [17]	*N*128; Gender: M66 F62; Age: 46.0 ± 12.1; UTP: 1.0–3.0 g/d.	*I* (*n* = 46): GTW (60 mg/d), irbesartan (300 mg/d).*C*1 (*n* = 42): GTW (60 mg/d). *C*2 (*n* = 40): irbesartan (300 mg/d). Follow-up period: 3 months.

Wei 2019 [18]	*N*70; Gender: *I*: M19 F16; *C*: M21 F14; Age: *I*: 39.57 ± 5.16; *C*: 37.65 ± 5.58.	*I* (*n* = 35): GTW (60 mg/d), irbesartan (150 mg/d). *C* (*n* = 35): irbesartan (150 mg/d). Follow-up period: 3 months.

Xu 2020 [19]	*N*58; Gender: *I*: M17 F12; *C*: M16 F13; Age: *I*: 39.65 ± 2.81; *C*: 40.03 ± 2.49	*I* (*n* = 29): GTW (30 mg/d), benazepril (10 mg/d). *C* (*n* = 29): benazepril (10 mg/d). Follow-up period: 3 months.

Feng 2020	*N*90; Gender: M57 F33; Age: 53.53 ± 9.52.	*I* (*n* = 45): GTW (60 mg/d), telmisartan (80 mg/d). *C* (*n* = 45): GTW (60 mg/d). Follow-up period: 3 months.

Wang, 2020 [21]	*N*34; Gender: *I*: M10 F7; *C*: M11 F6; Age: *I*: 42.61 ± 4.22; *C*: 43.75 ± 3.92.	*I* (*n* = 17): GTW (60 mg/d), olmesartan (20 mg/d). *C* (*n* = 17): olmesartan (20 mg/d). Follow-up period: 6 months.

Li and Huang, 2021 [22]	*N*110; Gender: *I*: M26 F29; *C*: M27 F28; Age: *I*: 41.52 ± 12.33; *C*: 41.47 ± 12.51.	*I* (*n* = 17): GTW (60 mg/d), telmisartan (40 mg/d). *C* (*n* = 17): telmisartan (40 mg/d). Follow-up period: 6 months

*Note. N*: number, M: male, F: female, *I*: intervention group, and *C*: comparison group.

**Table 2:** Definition of clinical outcomes in each study.

Studies	Complete remission (CR)	Partial remission (PR)	Total remission (TR)
Shen 2009 [10]	UTP < 0.3 g/d, ALB>35.0 g/L, Scr normal	UTP > 0.3 g/d, but reduced by more than 50% of the baseline value, renal function is stable (Scr < 25% baseline value)	CR and PR

Yu 2012 [11]	UTP reduced by ≥ 75%	UTP reduced by ≥ 50%, but ≤ 75%	CR and PR

Yang 2014 [12]	UTP reduced by ≥ 75%	UTP reduced by 50% ∼ 75%	CR and PR

Xiang 2014 [13]	UTP < 0.4 g/d, Scr normal	UTP is reduced by more than 50% of the baseline value, Scr rises by less than 50% of the base value	CR and PR

Yu 2016 [14]	UTP reduced by ≥ 75%	UTP reduced by 50% ∼ 75%	CR and PR

Zhu 2017 [15]	No introduction	No introduction	UTP reduced by ≥ 50%

Cai 2018 [16]	Macroscopic or microscopic hematuria basically disappear, and UTP is reduced by ≥ 80%	Macroscopic or microscopic hematuria improved significantly, and UTP was reduced by50%∼79%	CR and PR

Liang et al., 2019 [17]	UTP ≤ 0.3 g/d	UTP > 0.3 g/d, reduced by ≥ 50%	CR and PR

Wei 2019 [18]	UTP < 0.5 g/d, ALB > 30.0 g/L, clinical symptoms disappeared	UTP < 1.5 g/d, ALB: 25 ～ 30.0 g/L, improvement of clinical symptoms	CR and PR

Xu 2020 [19]	No introduction	No introduction	No introduction

Feng 2020 [20]	No introduction	No introduction	No introduction

Wang 2020 [21]	Complete disappearance of hematuria and proteinuria	Alleviation of hematuria and proteinuria symptoms	CR and PR

Li and Huang 2021 [22]	Symptoms disappear, no microscopic hematuria, UTP < 0.2 g/d	Symptoms improved significantly, with no microscopic hematuria, UTP < 0.2 g/d, reduced by >50%	CR and PR

**Table 3:** Reports of adverse events included in the study.

Studies	Therapeutic regimen	Sample size	Cough	Gastrointestinal symptoms	Elevated liver enzymes	Scr rise	WBC decline	Irregular menstruation	Dizziness headache	Skin allergies	Total
Shen 2009 [10]	GTW + Benazepril	26	4	0	2	0	3	0	0	0	9
	Benazepril	26	4	0	0	0	0	0	0	0	4

Yu 2012 [11]	GTW + Fosinopril	20	2	0	2	2	2	1	0	0	9
	Fosinopril	22	2	0	0	3	0	0	0	0	5

Yang 2014 [12]	GTW + Benazepril	32	0	2	0	0	1	0	0	0	3
	Benazepril	31	0	0	0	0	0	0	0	0	0
	TWM	33	0	2	0	0	0	0	0	0	2

Xiang 2014 [13]	GTW + Telmisartan	30	0	0	2	0	0	3	0	0	5
	Telmisartan	30	0	0	0	0	0	0	0	0	0

Yu 2016 [14]	GTW + Benazepril	30	?	?	?	?	?	?	?	?	?
	Benazepril	30	?	?	?	?	?	?	?	?	?
	GTW	30	?	?	?	?	?	?	?	?	?

Zhu 2017 [15]	GTW + ARB	30	0	0	5	0	0	0	0	0	5
	ARB	30	0	0	1	0	0	0	0	0	1

Cai 2018 [16]	GTW + Telmisartan	34	?	?	?	?	?	?	?	?	?
	Telmisartan	34	?	?	?	?	?	?	?	?	?

Liang et al., 2019 [17]	GTW + Irbesartan	46	0	2	0	0	0	0	0	0	2
	Irbesartan	40	0	2	0	0	0	0	0	0	2
	GTW	42	0	1	0	0	0	0	0	0	1

Wei 2019 [18]	GTW + Irbesartan	35	0	1	0	0	1	0	1	0	3
	Irbesartan	35	0	2	0	0	0	0	1	0	4

Xu 2020 [19]	GTW + Benazepril	29	?	?	?	?	?	?	?	?	?
	Benazepril	29	?	?	?	?	?	?	?	?	?

Feng 2020	GTW + Telmisartan	45	?	?	?	?	?	?	?	?	?
	GTW	45	?	?	?	?	?	?	?	?	?

Wang 2020 [21]	GTW + Olmesartan	17	?	?	?	?	?	?	?	?	?
	Olmesartan	17	?	?	?	?	?	?	?	?	?

Li and Huang 2021 [22]	GTW + Telmisartan	55	0	5	0	0	0	0	0	1	6
	Telmisartan	55	0	3	0	0	0	0	1	1	5

## Data Availability

The experimental data used to support the findings of this study are available from the corresponding author upon request.
